# The Application Value of Three-Dimensional Power Doppler Ultrasound in Fetal Growth Restriction

This article has been retracted.

**DOI:** 10.1155/2022/4087406

**Published:** 2022-08-16

**Authors:** Yanju Wang, Lihua Liang, Yingfeng Liu, Peipei Li, Jie Ren

**Affiliations:** ^1^Department of Ultrasound, The Fourth Hospital of Shijiazhuang, Shijiazhuang, Hebei, China; ^2^The Second Ward of Obstetrics, The Fourth Hospital of Shijiazhuang, Shijiazhuang, Hebei, China

## Abstract

In this study, the application value of three-dimensional power Doppler ultrasound (3D-PDU) in fetal growth restriction (FGR) is explored. The retrospective cohort study enrolled pregnant women (with a gestational week of 11–13 + 6 weeks) who received routine health care in the obstetrics and gynecology clinic of our hospital from January 2020 to January 2021. The placentae were scanned using 3D-PDU, and the subjects were followed up until delivery. The fetuses were divided into the control group (*n* = 322) and FGR group (*n* = 44) according to their birth weight. There was no significant difference in nuchal translucency (NT), crown-rump length (CRL), and placental volume (PV) during the first trimester between the two groups (*P* > 0.05). Compared with the control group, the FGR group showed significantly lower levels of vascularisation index (VI), flow index (FI), and vascularisation flow index (VFI) and a higher incidence of fetal distress and neonatal asphyxia (*P* < 0.05). The FGR group showed a longer gestational week at birth, a higher probability of cesarean section, and a lower 5-minute Apgar score than the control group (*P* < 0.05). The VI, FI, and VFI of the control group were significantly higher than those of the FGR group. Pearson analysis showed that birth weight was positively correlated with VI and FI (*P* < 0.05). 3D-PDU assesses the blood perfusion of the fetus and placenta in the first trimester and predicts the pregnancy outcome, which shows great potential in the early diagnosis of FGR.

## 1. Introduction

Fetal growth restriction (FGR), also known as intrauterine growth restriction (IUGR), accounts for about 30% of perinatal deaths and 50% of perinatal infants with intrauterine hypoxia during delivery, which is the second leading cause of perinatal deaths [1, 2]. FGR refers to a fetus of an abnormal size that does not reach its genetic growth potential in utero. Regardless of regional differences in the diagnostic criteria of FGR, the birth weight of the fetus is two standard deviations below the average weight for the same gestational week or 10% below the normal weight for the same gestational week [3]. Although the pathogenesis of FGR is still unclear, previous studies have revealed related influence factors, including maternal nutrition, placental transfer, and fetal genetic potential [4–6]. FGR is an important complication in the perinatal period that compromises the growth and development of the fetus and increases the morbidity of the fetus. Thus, early diagnosis and intervention is essential to achieve a better prognosis. However, FGR is usually diagnosed after delivery given the difficulty in the diagnosis of FGR in early pregnancy [7], which underscores the importance of accurate ultrasound examinations in the first trimester to dynamically assess fetal growth indicators [8]. Conventional two-dimensional ultrasound is a common method to assess FGR, but a reliable diagnosis of FGR is available at least after 27 weeks of gestation, with a limited capacity in evaluating placental circulation [9]. Three-dimensional power Doppler ultrasound (3D-PDU) combines three-dimensional ultrasound technology and power Doppler imaging and quantitatively evaluates the blood perfusion of the target tissue without interference by the detection angle and blood flow velocity, which is the current research hotspot of placental function evaluation [10]. To explore the value of 3D-PDU in the evaluation of FGR in the first trimester, this study performed 3D-PDU inspection on pregnant women admitted to the obstetrics and gynecology department of our hospital for routine health care from January 2020 to January 2021. The results are now reported as follows.

## 2. Materials and Methods

### 2.1. General Information

The retrospective cohort study enrolled pregnant women (11–13 + 6 weeks) who received routine health care in the obstetrics and gynecology clinic of our hospital from January 2020 to January 2021. The placentae were scanned using 3D-PDU and the participants were followed up until delivery. All study subjects underwent delivery or termination of pregnancy in our hospital. The fetuses were divided into the control group and FGR group according to their birth weight.

### 2.2. Inclusion Criteria

Pregnant women with a singleton pregnancy, clear last menstruation, regular menstruation, and normal uterine shape; with a clear gestational week of 11–13 + 6 weeks; with a 17 ≤ BMI ＜ 27 kg/m^2^; with communication ability and good treatment cooperation; and who provided written informed consent were included.

### 2.3. Exclusion Criteria

Pregnant women who had a fetus with fetal malformations or chromosomal abnormalities found during pregnancy or in the postpartum examination; with a height of <145 cm; with a previous negative pregnancy history such as stillbirth; and with uterine deformities were excluded. This study was approved by the Ethics Committee of the Fourth Hospital of Shijiazhuang, no. 20200058.

### 2.4. 3D-PDU Inspection

A Voluson 730 (GE Healthcare, Milwaukee, WI, USA) three-dimensional energy ultrasound diagnostic apparatus was used for scanning, with a frequency of 4.0–8.0 MHz of the volume probe, and VOCAL software was used for analysis. To avoid artifacts, the subjects were advised to maintain a calm breath and the fetus in a quiet state during the scanning. With the subject in a supine position, the fetal growth parameters were obtained with two-dimensional ultrasound. The 3D mode was used to predict whether the region of interest of the three-dimensional volume covers the entire placenta. The instrument parameters were adjusted according to the actual situation of the fetus, the noise was eliminated to a maximum extent, and the blood flow velocity in the placenta was maintained in the optimal state. During the inspection, an appropriate three-dimensional data box was used to ensure that the small villi vessels at the distal end of the placenta and the intact vascular tree from the base to the chorionic plate were completely displayed. The 3D-PDU of FGR placenta also showed the characteristics of 3D vascular tree, with fewer and thinner branches of the vascular tree than those of the normal group. After setting the angle, the placenta was continuously scanned for 15 s using the three-dimensional ultrasound probe in the PD mode to obtain the three-dimensional volume parameters of the placenta. Offline three-dimensional power Doppler and VOCAL software were used to measure and calculate the data. The placental volume (PV) was calculated by two experienced operators, and vascularisation index (VI), flow index (FI), and vascularisation flow index (VFI) were obtained from the software.

### 2.5. FGR Diagnostic Criteria

Fetuses with birth weight at delivery 10% below the normal birth weight of the same gestational week or a birth weight less than 2500 g after 37 weeks of gestation were diagnosed with FGR [3].

### 2.6. Observational Indicators

(1) The growth of the fetus: crown-lump length (CRL), nuchal translucency (NT), and placental volume (PV) were measured. The fetal's skull, brain midline, choroid plexus, four-chambered heart, gastric vesicle, bladder, umbilical cord insertion, limbs, and spine were monitored to rule out fetal malformations. (2) 3D-PDU indicators: 3D-PDU indicators include placental vascular function indexes such as VI, FI, and VFI. (3) Follow-up of newborns: all pregnant women gave birth in our hospital, and the gestational week, birth weight, delivery method, and Apgar score of newborns at birth were recorded.

### 2.7. Statistical Analysis

SPSS 22.0 was used for data analyses. The measurement data are expressed by (mean ± SD) and analyzed by the *t*-test. The counting data are expressed by (*n*%) and analyzed by the *χ*^2^ test. Pearson analysis was used for correlation analysis between neonatal weight and 3D-PDU indicators. The difference is considered statistically significant with *α* = 0.05.

## 3. Results

### 3.1. Comparison of the Baseline Data

A total of 366 cases of pregnant women were included in this study, including 44 cases of FGR pregnant women, with an incidence of 12.02% (44/366). As given in Table 1, the age of the pregnant women in the control group was 26.54 ± 5.36 years old, and the gestational week was 35.68 ± 5.25 weeks. There were 206 uniparae and 116 multiparae. The age of pregnant women in the FGR group was 27.06 ± 6.12 years, and the gestational week was 36.14 ± 4.07 weeks. There were 24 uniparae and 20 multiparae. The two groups presented no significant difference in baseline data (*P* > 0.05).

### 3.2. Comparison of Routine Screening Indicators in the First Trimester

As shown in Figure 1, in the control group, NT was 1.88 ± 0.55 mm, CRL was 75.36 ± 15.46 mm, and PV was 82.25 ± 25.36 cm^3^. The above indexes of the FGR group were 1.82 ± 0.46 mm, 71.29 ± 20.226 mm, and 78.29 ± 23.68 cm^3^, respectively. There was no significant difference in NT, CRL, and PV in the first trimester between the two groups (*P* > 0.05).

### 3.3. Comparison of 3D-PDU Indicators in the First Trimester

In the control group, VI was 20.36 ± 6.25%, FI was 48.21 ± 6.74, and VFI was 10.02 ± 2.19. The above indexes of the FGR group were 15.26 ± 5.29%, 43.15 ± 5.96, and 7.03 ± 2.34, respectively. The FGR group showed significantly lower VI, FI, and VFI levels than the control group (*P* < 0.05) (Table 2).

### 3.4. Comparison of Adverse Pregnancy Outcomes

All subjects in this study gave birth successfully. As given in Table 3, the control group had 22 cases of fetal distress and 6 cases of neonatal asphyxia, with the overall adverse reaction rate of 7.95% (28/322). The FGR group had 14 cases of fetal distress and 9 cases of neonatal asphyxia, with the overall adverse reaction rate of 31.82% (14/44). The incidences of fetal distress and neonatal asphyxia in the FGR group were significantly higher than those in the control group (*P* < 0.05).

### 3.5. Comparison of the Basic Conditions of Pregnant Women and Newborns

The FGR group had a longer gestational week at birth, a higher probability of cesarean section, and a lower 5-minute Apgar score of the birth weight than the control group (*P* < 0.05) (Table 4).

### 3.6. Relationship between 3D-PDU Indicators of Different Pregnancy Outcomes

According to the pregnancy outcome, the research subjects were divided into the normal pregnancy group (*n* = 334 cases) and the abnormal pregnancy group (*n* = 32 cases). The VI, FI, and VFI of the control group were significantly higher than those of the FGR group (*P* < 0.05) (Table 5).

### 3.7. Correlation Analysis of Birth Weight and 3D-PDU Indicators

As given in Table 6, birth weight was positively correlated with VI (*r* = 0.692, *P*=0.006) and FI (*r* = 0.526, *P*=0.024). There was no significant correlation between birth weight and VFI.

## 4. Discussion

In the present study, there was no significant difference in the NT, CRL, and PV of the fetus in the first trimester between the two groups [11]. Compared with the control group, the FGR group showed a higher incidence of fetal distress and neonatal asphyxia (*P* < 0.05). Moreover, the FGR group had a longer gestational week at birth, a higher probability of cesarean section, and a lower 5-minute Apgar score of the birth weight than the control group. FGR is closely related to the risk of adverse perinatal outcomes, including fetal death, low Apgar score, oligohydramnios, placental abruption, and neonatal critical illness [12].

Traditional ultrasound detection assesses fetal weight after 27 weeks of gestation based on biometrics, but the diagnostic accuracy is considered poor for FGR. The effectiveness of traditional Doppler ultrasound in evaluating placental function is confronted with the following problems. The placenta is an organ with relatively low resistance and slow blood flow. Color Doppler ultrasound can neither detect the low-speed blood flow inside the placenta villi space nor identify the individual villi blood vessels [13]. Several large cohort studies have also indicated that conventional ultrasound changes are associated with low sensitivity and specificity in the FGR population [14]. FGR is mostly caused by placental dysfunction secondary to uterine-placental-fetal blood circulation disorders, and early diagnosis is of great significance for its treatment and prognosis [15]. Placental function assessment is to understand the state of blood circulation and material exchange between mother and fetus, which contributes to assessing the developmental status of the fetus. However, the ultrasound imaging of the placenta is rather unsatisfactory in the first trimester. 3D-PDU showed a high sensitivity in visualization of villous blood vessels in placenta and even distal branches, providing information about vascular density, diameter change, and curvature and calculating three vascular indexes such as VI, FI, and VFI in the form of a histogram to achieve the quantitative evaluation of blood vessel density and blood perfusion in the placenta [16].

Herein, the VI, FI, and VFI of the FGR group were significantly lower than those of the control group, indicating a high predictive value of 3D-PDU in the first trimester. VI, FI, and VFI are the main indicators of 3D-PDU, which are closely related to the real blood vessel density and blood perfusion in the placenta and are available for objective and quantitative analysis [17]. A previous research has confirmed the negative impact of FGR on the blood supply to the placenta. Specifically, abnormalities of the villi vessels in the placenta initiates the remodeling compensatory response of the vascular wall, increasing the content of collagen and elastin and reinforcing the hardness of the blood vessels, which results in the increase of placental vascular resistance and reduction of the placental perfusion [18]. Another study has stated that FGR was related to uterine spiral artery remodeling during pregnancy, causing placental plaque necrosis, reduction or disappearance of villi vessels, and placental dysfunction [19].

Pearson analysis in the present study showed that birth weight was positively correlated with VI and FI (*r* = 0.692, 0.526), which is consistent with the results of a prior study which suggested that the 3D-PDU indexes are linearly positively correlated with fetal body mass and positively correlated with fetal double parietal diameter, head circumference, abdominal circumference, femoral length, and double occipital diameter [20]. Furthermore, in the present study, the correlation coefficient between FI and birth weight was less than VI, which may be attributed to the impact of placental blood vessels and uterine and umbilical artery on FI. Limitations of this study lie in the following aspects. First, this study did not continuously observe the continuous dynamic changes of 3D-PDU and fails to determine the trend of 3D-PDU indicators with the gestational week and the reference range of different gestational weeks. Moreover, 3D-PDU has more stringent requirements for ultrasound machines and radiologists. Therefore, its clinical application feasibility requires further verification.

## 5. Conclusions

3D-PDU assesses the blood perfusion of the fetus and placenta in the first trimester and predicts the pregnancy outcome, which shows great potential in the early diagnosis of FGR.

## Figures and Tables

**Figure 1:** Comparison of routine screening indicators in the first trimester. (a) NT. (b) CRL. (c) PV.

**Table 1:** Comparison of baseline data of two groups of pregnant women.

	Control group (*n* = 322)	FGR group (*n* = 44)	*t*/*χ*^2^	*P*
Age	26.54 ± 5.36	27.06 ± 6.12	1.147	0.252
Gestational age	35.68 ± 5.25	36.14 ± 4.07	0.459	0.647
Primipara	206	24	1.474	0.225
Tobacco use	42	8	0.867	0.352
Alcohol exposure	59	9	0.116	0.733
Chronic hypertension	46	6	0.013	0.908
Pregestational diabetes	28	7	2.329	0.127

**Table 2:** Comparison of 3D-PDU indicators in the first trimester between the two groups of pregnant women.

	VI	FI	VFI
Control group (*n* = 322)	20.36 ± 6.25	38.21 ± 6.74	8.02 ± 2.19
FGR group (*n* = 44)	15.26 ± 5.29	33.15 ± 5.96	6.03 ± 2.34
*t*	5.164	4.732	5.607
*P*	<0.001	<0.001	<0.001

**Table 3:** Comparison of adverse pregnancy outcomes between the two groups of pregnant women.

	Fetal distress	Neonatal asphyxia	Total incidence
Control group (*n* = 322)	12	6	18
FGR group (*n* = 44)	9	5	14
*χ* ^2^	20.03	11.99	33.38
*P*	<0.001	<0.001	<0.001

**Table 4:** Comparison of the basic conditions of the two groups of pregnant women and newborns.

	Control group (*n* = 322)	FGR group (*n* = 44)	*t*/*χ*^2^	*P*
Gestational age at birth	36.25 ± 2.52	39.95 ± 2.67	9.070	<0.001
Delivery mode			10.02	0.002
Vaginam cesarean delivery	269	28		
Cesarean delivery	53	16		
5-minute apgar scores	9.26 ± 1.58	7.11 ± 2.75	7.604	<0.001
Birth weight, g	2598 ± 659	3016 ± 642	3.958	<0.001

**Table 5:** Relationship between 3D-PDU indicators of pregnant women with different pregnancy outcomes.

	VI	FI	VFI
Normal pregnancy (*n* = 334)	22.59 ± 5.16	37.59 ± 4.06	9.28 ± 2.15
Bad pregnancy (*n* = 32)	14.29 ± 4.59	29.25 ± 3.69	5.22 ± 1.68
*t*	8.771	11.18	10.38
*P*	<0.001	<0.001	<0.001

**Table 6:** Correlation analysis of birth weight and 3D-PDU index.

	Birth weight	
	*r* (95% CI)	*P*
VI	0.692 (0.512, 0.732)	0.006
FI	0.526 (0.471, 0.673)	0.024
VFI	0.321 (0.274, 0.432)	0.079

## Data Availability

The data used to support the findings of this study are available from the corresponding author upon request.

## References

[1] Nardozza L. M., Caetano A. C., Zamarian A. C. (2017). Fetal growth restriction: current knowledge. *Archives of Gynecology and Obstetrics*.

[2] Gordijn S. J., Beune I. M., Thilaganathan B. (2016). Consensus definition of fetal growth restriction: a Delphi procedure. *Ultrasound in Obstetrics and Gynecology*.

[3] Salomon L. J., Alfirevic Z., Da Silva Costa F. (2019). ISUOG Practice Guidelines: ultrasound assessment of fetal biometry and growth. *Ultrasound in Obstetrics and Gynecology*.

[4] Audette M. C., Kingdom J. C. (2018). Screening for fetal growth restriction and placental insufficiency. *Seminars in Fetal and Neonatal Medicine*.

[5] Colella M., Frérot A., Novais A. R. B., Baud O. (2018). Neonatal and long-term consequences of fetal growth restriction. *Current Pediatric Reviews*.

[6] Borrell A., Grande M., Pauta M., Rodriguez-Revenga L., Figueras F. (2018). Chromosomal microarray analysis in fetuses with growth restriction and normal karyotype: a systematic review and meta-analysis. *Fetal Diagnosis and Therapy*.

[7] Figueras F., Gratacós E. (2014). Update on the diagnosis and classification of fetal growth restriction and proposal of a stage-based management protocol. *Fetal Diagnosis and Therapy*.

[8] Baschat A. A. (May 2018). Planning management and delivery of the growth-restricted fetus. *Best Practice and Research Clinical Obstetrics and Gynaecology*.

[9] Luria O., Barnea O., Shalev J. (2012c). Two-dimensional and three-dimensional Doppler assessment of fetal growth restriction with different severity and onset. *Prenatal Diagnosis*.

[10] Noguchi J., Hata K., Tanaka H., Hata T. (May 2009). Placental vascular sonobiopsy using three-dimensional power Doppler ultrasound in normal and growth restricted fetuses. *Placenta*.

[11] Kennedy L. M., Tong S., Robinson A. J. (2020). Reduced growth velocity from the mid-trimester is associated with placental insufficiency in fetuses born at a normal birthweight. *BMC Medicine*.

[12] Molina L. C. G., Odibo L., Zientara S. (2020). Validation of Delphi procedure consensus criteria for defining fetal growth restriction. *Ultrasound in Obstetrics and Gynecology*.

[13] Tanaka H., Furuhashi F. H., Toriyabe K. (2019). Management of fetal growth restriction using the contraction stress test: a case-control study. *Journal of Maternal-Fetal and Neonatal Medicine*.

[14] Zhang N., Schumacher A., Fink B., Bauer M., Zenclussen A. C., Meyer N. (2022). Insights into early-pregnancy mechanisms: mast cells and chymase CMA1 shape the phenotype and modulate the functionality of human trophoblast cells, vascular smooth-muscle cells and endothelial cells. *Cells*.

[15] Zur R. L., Kingdom J. C., Parks W. T., Hobson S. R. (2020). The placental basis of fetal growth restriction. *Obstetrics and Gynecology Clinics of North America*.

[16] Abdallah A., Khairy M., Tawfik M. (2021). Role of first-trimester three-dimensional (3D) power Doppler of placental blood flow and 3D placental volume in early prediction of pre-eclampsia. *International Journal of Gynecology and Obstetrics*.

[17] Noguchi J., Tanaka H., Koyanagi A., Miyake K., Hata T. (2015). Three-dimensional power Doppler indices at 18–22 weeks’ gestation for prediction of fetal growth restriction or pregnancy-induced hypertension. *Archives of Gynecology and Obstetrics*.

[18] Nugent J. L., Wareing M., Palin V. (2013). Chronic glucocorticoid exposure potentiates placental chorionic plate artery constriction: implications for aberrant fetoplacental vascular resistance in fetal growth restriction. *Endocrinology*.

[19] Lyall F., Robson S. C., Bulmer J. N. (2013). Spiral artery remodeling and trophoblast invasion in preeclampsia and fetal growth restriction: relationship to clinical outcome. *Hypertension*.

[20] Bozkurt N., Başgül Yigiter A., Gokaslan H., Kavak Z. N. (2010). Correlations of fetal-maternal outcomes and first trimester 3-D placental volume/3-D power Doppler calculations. *Clinical and Experimental Obstetrics and Gynecology*.

